The article "CT Image Analysis and Clinical Diagnosis of New Coronary Pneumonia Based on Improved Convolutional Neural Network" was published in 2021. Journal: Comput Math Methods Med.

# CT Image Analysis and Clinical Diagnosis of New Coronary Pneumonia Based on Improved Convolutional Neural Network

**DOI:** 10.1155/2021/7259414

**Published:** 2021-07-20

**Authors:** Wu Deng, Bo Yang, Wei Liu, Weiwei Song, Yuan Gao, Jia Xu

**Affiliations:** ^1^College of Electronic Information, Sichuan University, Chengdu Sichuan 610000 ., China; ^2^Information Center/Engineering Research Center of Medical Information Technology, Ministry of Education, West China Hospital of Sichuan University, Chengdu Sichuan 610000, China; ^3^Information Center/Engineering Research Center of Medical Information Technology, West China Hospital of Sichuan University, Chengdu Sichuan 610000, China; ^4^Department of Radiology, West China Hospital of Sichuan University, Chengdu Sichuan 610000, China; ^5^College of Physics, Sichuan University, Chengdu Sichuan 610000, China

## Abstract

In this paper, based on the improved convolutional neural network, in-depth analysis of the CT image of the new coronary pneumonia, using the U-Net series of deep neural networks to semantically segment the CT image of the new coronary pneumonia, to obtain the new coronary pneumonia area as the foreground and the remaining areas as the background of the binary image, provides a basis for subsequent image diagnosis. Secondly, the target-detection framework Faster RCNN extracts features from the CT image of the new coronary pneumonia tumor, obtains a higher-level abstract representation of the data, determines the lesion location of the new coronary pneumonia tumor, and gives its bounding box in the image. By generating an adversarial network to diagnose the lesion area of the CT image of the new coronary pneumonia tumor, obtaining a complete image of the new coronary pneumonia, achieving the effect of the CT image diagnosis of the new coronary pneumonia tumor, and three-dimensionally reconstructing the complete new coronary pneumonia model, filling the current the gap in this aspect, provide a basis to produce new coronary pneumonia prosthesis and improve the accuracy of diagnosis.

## 1. Introduction

Novel coronavirus pneumonia (NCP) is referred to as novel corona pneumonia, which refers to pneumonia caused by 2019 novel coronavirus infection (2019 Novel Coronavirus (COVID-19)) [1]. Since December 2019, Wuhan City, Hubei Province, has successfully discovered multiple cases of NCP patients with COVID-19 infection [2]. Coronavirus is a type of RNA virus with an envelope and a linear single-stranded genome. Obvious rod-shaped particles are protruding on the shape of the corolla, so it is named coronavirus [3]. Coronavirus only infects vertebrates and is related to a variety of diseases in humans and animals. It can cause respiratory and digestive tract and nervous system diseases in humans and animals. So far, in a total of 7 coronaviruses that can infect humans, 3 coronaviruses can cause severe respiratory diseases, namely COVID-19, SARS-CoV, and MERS-CoV, respectively. The early manifestations are mainly patchy ground-glass shadows in the double lungs [4]. As the lesion progresses, the lesions increase with consolidation, and bronchial inflation signs, “paving stone signs,” “halo signs,” and “antihalo signs” may occur. The lungs are diffusely real. During the recovery period, the lung lesions are absorbed and fibrous foci formed, and there were less hilar and mediastinal lymphadenopathy and a large amount of pleural effusion [5]. Because deep learning methods are more efficient in analyzing images, the results are more accurate.

The article "CT Image Analysis and Clinical Diagnosis of New Coronary Pneumonia Based on Improved Convolutional Neural Network" was published in 2021. Journal: Comput Math Methods Med.

The semantic segmentation of an image is to classify pixels according to the category to which the pixels belong, divide pixels belonging to the same category, and then realize image segmentation [6, 7]. The segmentation algorithm based on the texture primitive forest combines the context information of the image, expresses the image as a histogram distribution of the texture image, to train the *K*-nearest neighbor or support vector machine classifier, and then classifies the image to achieve the purpose of image segmentation [8]. However, this algorithm is greatly affected by the changes in illumination and image rotation in the neighborhood [9]. Different neighborhood sizes have different classification performance, and different images will have different optimal neighborhood sizes [10]. The segmentation method based on random forest directly uses the low-level pixels of the image, extracts a fixed-size window from the image to obtain a feature vector according to random sampling, and then randomly selects two pixels from the window to obtain the value vector, training random forest classifier [11]. The specific method is to vote for the vector extracted from each window through the leaf nodes of the random forest, predict the pixel type according to the voting result, and complete the semantic segmentation of the image [12]. In contrast, this method can greatly improve the segmentation efficiency. In the early deep learning methods, the classification network usually has a fully connected layer whose input is a fixed-size pixel block [13]. Therefore, the semantic segmentation applied to the image classified based on image block 3, that is, the pixels around each pixel extracted from the image. The image block is composed and used to judge the category of the pixel [14]. Not only this segmentation algorithm is cumbersome to calculate but also the effect is not ideal [15]. In 2017, at the University of California, Jiang and others proposed a fully convolutional neural network (FCN) to change the fully connected layer in the previous convolutional neural network to a convolutional layer [16]. FCN does not require a fully connected layer to perform dense pixel prediction and can accept input images of any size while avoiding the problem of repeated storage and calculation convolution caused by using pixel blocks, which accelerates the processing speed and is more efficient [17]. Therefore, the neural network for semantic segmentation mostly adopted the structure of FCN. The appearance of FCN is a milestone for the application of a convolutional neural network to image semantic segmentation [18]. Based on the FCN network structure, Mazurowski et al. proposed a 3D FCN for segmentation of a new type of coronary pneumonia MRI image and further optimized the segmentation results through the deformation model algorithm to improve the accuracy of image segmentation [19]. Pan et al. first used CT images to train the 2D FCN network, input the CT images of the sagittal plane, coronal plane, and cross-section corresponding to each pixel, and then used the 3D majority-voting algorithm to perform the three-image vote on the segmentation result to obtain the final segmentation result [20]. Pons and others input the coronary MRI images in brain MRI, myocardial MRI, and cardiac CT angiography into the same FCN network, so that the final trained network can perform the segmentation tasks for the above three types of images at the same time [21].

The article "CT Image Analysis and Clinical Diagnosis of New Coronary Pneumonia Based on Improved Convolutional Neural Network" was published in 2021. Journal: Comput Math Methods Med.

This article focuses on the research of the new coronary pneumonia tumor image diagnosis method. Through deep learning and preoperative new coronary pneumonia tumor CT images, the new coronary pneumonia tumor image automatic segmentation, tumor detection, and diagnosis will assist doctors in preoperative tumor identification and diagnosis, and follow-up. The main research contents of this article include segmentation of the vertebral body area and surrounding soft tissues in the CT image of the new coronary pneumonia, detection, and identification of tumor lesions of the new coronary pneumonia, and image diagnosis of the new coronary pneumonia. In this paper, firstly, the CT image of the new coronary pneumonia is segmented by the convolutional neural network, and the new coronary pneumonia area is extracted to obtain the binary image with the new coronary pneumonia area as the foreground and the remaining areas as the background. The convolutional neural network has a strong feature learning ability. Then, based on the deep convolutional neural network, feature extraction is performed on the new type of coronary pneumonia tumor image to obtain a higher-level abstract representation of the feature and then predict the lesion location and obtain its bounding box in the image. Finally, by generating an adversarial network for image diagnosis of the CT image of the new coronary pneumonia tumors, the normal new coronary pneumonia CT image output network is trained to obtain the corresponding network model, and then the tumor area in the CT image of the new coronary pneumonia tumor is added, the mask is used as the input of the model, and the output of the model is the image of the complete new coronary pneumonia diagnosed. The image after the diagnosis will be used to reconstruct the complete three-dimensional digital model of the new coronary pneumonia through a three-dimensional reconstruction algorithm, which provides a basis for the subsequent production of the new coronary pneumonia.

The article "CT Image Analysis and Clinical Diagnosis of New Coronary Pneumonia Based on Improved Convolutional Neural Network" was published in 2021. Journal: Comput Math Methods Med.

## 2. CT Image Analysis of New Coronary Pneumonia Based on Convolutional Neural Network

### 2.1. Improved Convolutional Neural Network Model

The traditional medical image segmentation methods used in this paper include region-based segmentation methods, such as threshold method, region growth algorithm, and level set-based segmentation methods. The threshold segmentation algorithm is the most common image segmentation method [22]. The algorithm assumes that the pixel values of the adjacent pixels in the target or background in the gray image are similar, but the pixel values of different targets are different. In the results presented on the image histogram, different targets correspond to different peaks, so the threshold at the peak and valley positions is selected to separate the different targets. In turn, the lesion site is predicted, and its bounding box in the image is obtained. Finally, the image diagnosis of the novel coronary pneumonia tumor CT images is performed by generating an adversarial network, and the normal novel coronary pneumonia CT images are output to the network for training to obtain the corresponding network model. If only one threshold is selected, the image is divided into a single target area and a background area, which is called single threshold segmentation; if multiple thresholds are selected, the image is divided into multiple target areas, which is called multithreshold segmentation. The advantage of this method is that it is relatively simple to implement. When the gray values of different categories are very different from other feature values, the image can be effectively segmented; accordingly, if the gray difference in the image is not large or the gray between regions the value ranges overlap, it is difficult for the algorithm to segment accurate results. The basic idea of the area growth algorithm is to gather pixels with similar properties: first, select a seed point and then traverse the pixels in the image, in turn, to determine the pixels about the seed [23]. If the similarity is satisfied, it is divided into seed areas at the same time, and the pixel is pushed into the stack as an alternative seed point until all pixels have a home and eventually form a different area. The algorithm is simple to calculate and particularly suitable for segmenting small structures, such as tumors and scars. The point has great impact on the segmentation results and is sensitive to noise, as shown in Figure 1.

The article "CT Image Analysis and Clinical Diagnosis of New Coronary Pneumonia Based on Improved Convolutional Neural Network" was published in 2021. Journal: Comput Math Methods Med.

Since the introduction of ResNet, it has proved that increasing the number of network models and the accuracy of the model can be considered. Therefore, there are endless variations of the network, and the improved model further improves performance. The 2017 CVPR best paper DenseNet also draws on the idea of ResNet and at the same time creatively proposed a brand-new structure. DenseNet is a densely connected convolutional neural network [24]. Like ResNet, the model contains multiple dense blocks. There are connections between any two layers. Specifically, each layer of input is all previous layers. The union of the output of the feature map extracted by this layer will also directly be passed to the subsequent convolutional layer. The purpose of this is to ensure that the information flow between the layers reaches the maximum.

Unlike the ResNet model, the elements between the layers added together and the connection between the different layers in DenseNet are splicing, which is the superposition of dimensions. This dense connection method will reduce the computational cost of each layer of the network and will reuse features. There is no need to relearn redundant feature maps. The operation of dimensional stitching will add more features, compared with the model [25]. Another advantage of DenseNet is that the configuration of its structure allows each layer to directly obtain gradients from the loss function and model input, which improves the flow of information and gradients in the model, which is very beneficial for training. In ResNet, due to the residual learning module, the output of the *u* layer can be expressed as

(1) $$\begin{array}{c} -\mathrm{div}\left(\frac{\nabla^{a}u}{\left|\nabla^{a}u\right|+p}\right)+\lambda_{e}\left(u-u^{0}\right)=0. \end{array}$$

The identity map and the output of the nonlinear transformation superimposed in an additive manner, which destroys the information flow in the model to a certain extent. However, in DenseNet, the output of layer *X* can be expressed as

(2) $$\begin{array}{c} \left(a,b;X,\Phi \right)={\left|a\right|}^{-0.5}\int_{-\propto }^{+\propto }a\left(\tau \right)g\left(\tau -t\right)e^{-jw\tau }d\tau . \end{array}$$

According to the definition of migration learning, migration learning can be divided into three types, distribution difference migration learning, feature difference migration learning, and label difference migration learning. Distribution difference migration learning has different edge distribution or conditional probability distribution for source and target domain data, feature difference migration learning has different feature space for source and target data, and label difference migration learning refers to different data tagging space for source and target domains. Since each layer contains the output information of all previous layers, only a few feature maps are needed. It is enough and can reduce the phenomenon of gradient disappearance. When tensor stitching, the size of the feature map needs to be the same; otherwise, the dimensions cannot be superimposed. However, pooling operation is essential. To reconcile this contradiction, DenseNet adds a transition layer between dense blocks.

The article "CT Image Analysis and Clinical Diagnosis of New Coronary Pneumonia Based on Improved Convolutional Neural Network" was published in 2021. Journal: Comput Math Methods Med.

The loss function in the original *K*_*nn*_ is

(3) $$\begin{array}{c} k_{nn}\left(x\right)=\overset{N}{\underset{i=1}{\sum }}w_{i}s_{i}\left(x\right)=W^{T}S\left(x\right). \end{array}$$

The first term does not depend on the generator and can be used as a generator loss function. However, for the discriminator, the generator is optimized by fixing the generator, and the contribution to the discriminator loss function is

(4) $$\begin{array}{c} D_{\varepsilon }\left(x\left(t\right)\right)=\left[s\left(\left\|x\left(t\right)-\ell_{j1}\right\|\right)\right]. \end{array}$$

The data is then randomly assigned. Since the discriminator in formula (4) maximizes the loss function on the right, it is added with a minus sign and converted to find the minimum value, so that it derives about the *Q*_*N*_(*w*) pair:

(5) $$\begin{array}{c} Q_{N}\left(w\right)=\frac{1}{2}\underset{i,j}{\sum }P_{ij}{\left(1-P_{ij}\right)}^{2}+{\left\|w^{T}X_{b}\right\|}_{2}^{2}. \end{array}$$

Get the optimal discriminator function:

(6) $$\begin{array}{c} \phi_{m,n}=\frac{{\left\|q_{m,n}\right\|}^{2}}{\delta^{2}}\exp\left(-\frac{\left(q_{m,n}*z\right)}{2\delta^{2}}\right)*\left[e^{i\left(q_{m,n}*z\right)}-e^{-\delta^{2}/2}\right]. \end{array}$$

Intuitively, formula (4) represents the relative proportion of sample *x* from the true distribution and the probability of generating distribution, and it is substituted into formula (2):

(7) $$\begin{array}{c} \frac{\partial L}{\partial a}=\overset{n}{\underset{i=1}{\sum }}\left[y_{i}-\frac{\exp\left(a+\sum_{j=1}^{m}x_{ij}\beta_{j}\right)}{1+\exp\left(a+\sum_{j=1}^{m}x_{ij}\beta_{j}\right)}\right]=0. \end{array}$$

It can be further transformed into

(8) $$\begin{array}{c} \frac{\partial L}{\partial \beta_{j}}=\overset{n}{\underset{i=1}{\sum }}\left[y_{i}-\frac{\exp\left(a+\sum_{j=1}^{m}x_{ij}\beta_{j}\right)}{1+\exp\left(a+\sum_{j=1}^{m}x_{ij}\beta_{j}\right)}x_{ij}\right]=0,j=1,2,.\cdots ,m,\\ g_{i}=\omega_{i}/\overset{n}{\underset{j=1}{\sum }}\omega_{i},\overset{n}{\underset{i=1}{\sum }}g_{i}=1. \end{array}$$

Divergence is as follows:

(9) $$\begin{array}{c} b_{ij}=\frac{b_{ij}}{\sum_{k=1}^{n}b_{kj}\left(i,j=1,2,\cdots n\right)}. \end{array}$$

The development of medical image segmentation technology not only affects the development of other related technologies in medical image processing, such as visualization and 3D reconstruction, but also occupies an extremely important position in the analysis of biomedical images. In recent years, medical image segmentation techniques have made remarkable progress due to the application of some emerging disciplines in medical image processing. In this paper, we take the perspective of the specific theoretical tools applied for segmentation. As can be seen from the above derivation formula, when the training discriminator is close to the optimal, the divergence will be smaller, but when there is no overlap between the real distribution and the generated distribution or the overlapping part can be ignored, the JS divergence will be fixed and constant, which means that the gradient is zero. Therefore, when the discriminator is in the optimal situation, the generator cannot obtain the gradient information, which results in unstable training. *b* replaces *P* divergence with the Wasserstein distance to measure the distance between the real distribution and the generated distribution, which is defined as follows:

(10) $$\begin{array}{c} P\left(y_{i}\right)=p_{i}^{y_{i}}{\left(1-p_{i}\right)}^{1-y_{i}}. \end{array}$$

Since the lower bound value in formula (10) cannot be solved directly, it is transformed into

(11) $$\begin{array}{c} m=P\left(R\left|S\right.\right)=\frac{P\left(S\cap M\right)}{P\left(S\right)}=\frac{s}{s+h}. \end{array}$$

The article "CT Image Analysis and Clinical Diagnosis of New Coronary Pneumonia Based on Improved Convolutional Neural Network" was published in 2021. Journal: Comput Math Methods Med.

### 2.2. Design of CT Image Dataset for New Coronary Pneumonia

Before training the network, it is necessary to make a new type of coronary pneumonia CT image data set and corresponding annotation data. First, for the original image, you need to convert its format to the BMP or jpg format required by this article, remove the patient's information data from the original image, and then use the traditional segmentation method, that is, the above level set to process the original new coronary pneumonia CT. We perform segmentation to obtain labeled data and divide the data set into a training set and a test set according to a 7 : 3 ratio. This may lead to a high false-positive rate of 27.49% in the LIDC-IDRI dataset for physicians with benign and malignant lung nodules. Besides, the training process will be verified by a 10-fold cross-validation method. Ten-fold cross-validation is to divide all the training sets into ten parts, take one of them for testing without repeating each time, which is the so-called verification set, and use the other nine parts as training sets to train the model. Before training the network, this paper needs to enhance the data of the new coronary pneumonia CT image, which on the one hand increases the amount of data and, on the other hand, is conducive to the network's adaptability to tissue deformation. The process of data enhancement is shown in Figure 2. After using the level set method to segment the new coronary pneumonia CT image to obtain the label, the training set and the corresponding label are channel merged, then the merged image is subjected to such as rotation, translation, and image processing such as mirroring, so that the training set image and the corresponding label get the same transformation, and finally, the transformed combined image is separated into the training set and the label, thereby obtaining the expanded training set and the corresponding label.

Due to the outstanding performance of U-Net in medical image segmentation tasks, this paper will complete the segmentation task of new-type coronary pneumonia CT images through this type of network. U-Net is a typical end-to-end network structure. As its name indicates, its structure is U-shaped. Aiming at the task of new-type coronary pneumonia CT image segmentation in this paper, some adjustments were made to the original U-Net, as shown in Figure 3. The entire network is divided into two processes. The first is the downsampling process, which is used to capture context information. Four sets of convolution operations are completed. After each set of convolution operations, the feature map is pooled to reduce the image to half of the original after four convolution operations, and the original image with the original size of 512 × 512 is reduced to 16 × 16. Then, there is the upsampling process, which also uses four sets of deconvolution operations. Each upsampling expands the size of the feature map to twice the original size and stitches with the corresponding feature map during the downsampling process. The size is 256 × 256 × 16 feature map. Finally, the number of channels is reduced to 1 by a 1 × 1 convolution kernel. Its specific parameters are shown in Figure 3. In the downsampling process, this paper uses a convolution kernel of size 9 × 9 and padding to perform the convolution operation. The advantage of this is that the feature maps at each stage of upsampling have the same resolution, and upsampling and downsampling corresponding to the size of the feature map are the same, eliminating the cropping operation during splicing, and can retain all the information extracted by the convolution operation.

The article "CT Image Analysis and Clinical Diagnosis of New Coronary Pneumonia Based on Improved Convolutional Neural Network" was published in 2021. Journal: Comput Math Methods Med.

V-Net is a further improvement based on U-Net, which is used to segment three-dimensional data. Since the problem to be solved in this article is the segmentation of two-dimensional images, we will extract the core elements in V-Net to complete the new crown pneumonia CT image segmentation task. The encoder-decoder structure is like U-Net, except that the input and output of the convolutional layer in each stage of the encoder are added to obtain residual learning. The result of this is to be able to retain due to compress the lost information, improve the accuracy of the target boundary segmentation in the image, converge in a short time, and improve the model convergence speed. The basic idea of the region growing algorithm is to merge pixel points with similar properties together. For each region, a seed point is designated as the starting point for growth, then the pixels in the field around the seed point are compared with the seed point, and the points with similar properties are merged and continue to grow outward until no pixels that meet the conditions are included. In this way, the growth of a region is completed. And in the encoder, after each stage of the feature map processing, the resolution will be compressed by the convolution kernel of 4 × 4 and step size 4, thereby achieving the effect of reducing the size of the feature map to half, which is like the function of the pooling operation that not only does not lose edge information but also does not need to switch the mapping between input and output in the pooling operation, which reduces the use of memory. At the same time, in the entire network, the size of the convolution kernel in each stage of the convolution operation is 10 × 10, and the PReLU nonlinear activation function is used.

### 2.3. Analysis and Diagnostic Evaluation Design

The main purpose of fine-grained classification is to distinguish multiple subcategories under the same basic category. Each subcategory shares very similar attribute characteristics, and the differences between subcategories are very subtle, so fine-grained classification is very challenging. In the medical background, there are few studies on the problem of fine-grained image analysis, which is mainly due to the exploration of fine-grained medical image analysis that is limited by the existing data and annotations. Data labeling requires professional knowledge, and the cost of labeling is very expensive. However, the fine-grained evaluation will bring about a reduction in the sample of each subclass of the attribute and a more subtle difference in its characteristics. At the same time, the samples of each subclass are extremely unbalanced. As shown in Table 1, the distribution is very biased. The slanted situation and the lack of coverage of minority samples will cause the algorithm to have serious problems in the underrepresented minority classes. The problem of data imbalance in the fine-grained attribute subclasses of lung nodules can easily bias the learning framework. This further increases the difficulty of fine-grained medical image analysis. Traditional oversampling techniques implicitly assume that the behavior of oversampling will not deviate from the original class distribution. However, this assumption does not apply to complex high-dimensional data, because the synthetic samples of these data are inherently difficult, and simple interpolation can easily deviate from the original class distribution.

The article "CT Image Analysis and Clinical Diagnosis of New Coronary Pneumonia Based on Improved Convolutional Neural Network" was published in 2021. Journal: Comput Math Methods Med.

In the experiment, we implemented 5 network models based on the network structure shown in Figure 3. Basic network, where*n*_1_,*n*_2_, and*n*_3_are 32, 64, and 128 and 64, 128, and 256, respectively, and the model, where*n*_1_,*n*_2_, and*n*_3_are 64, 128, and 256, use bounce connection, only residual learning, and both. The initial learning rate is set to 0.001, the learning rate decays to the original 0.2 every 50 cycles, and a total of 200 cycles are trained to obtain the final model of each network. Then, we calculate the average of the SSIM and PSNR indicators of the 40 chest radiographs of the test set and the DES label. The model and corresponding evaluation results are shown in Figure 4. Both PSNR and SSIM are larger. The higher the similarity between the two images, the experimental data shows that both bounce connection and residual learning can improve the performance of the model. If used simultaneously, the model is better. Also, the network's increased number of convolution cores can improve the performance. Both PSNR and SSIM indicate that the larger the value, the higher the similarity between the two images. Experimental data shows that both bounce connection and residual learning can improve the performance of the model. If used simultaneously, the model is better. Besides, the network's increased number of convolution cores can also improve the performance.

The article "CT Image Analysis and Clinical Diagnosis of New Coronary Pneumonia Based on Improved Convolutional Neural Network" was published in 2021. Journal: Comput Math Methods Med.

During preprocessing, the original image is first scaled to a resolution of 1024 × 1024, which is consistent with the resolution used by the model during training, and then the coordinate values of the nodule annotations are adjusted accordingly. Although the fully convolutional network does not require that the input image size must be the same, because our training data is relatively small and the source is single, to reduce the model's “unfit” on the new data, we adjusted the new chest radiograph image that is consistent with the input image resolution when the skeleton suppression model is trained. After these images were processed by the rib suppression network, and then the size was converted to the original size, the ribless chest radiograph data was obtained. Then, we used the target-detection network RetinaNet as the detection model to verify the effect of our proposed rib suppression method on the detection of lung nodules on 5908 chest radiographs with lung nodules. We randomly selected 296 chest radiographs as the test set and the remaining 5612 samples as the training set. The two data sets were divided the same, and the image size was adjusted to 1024 × 1024. The anchor aspect ratio in RetinaNet is [0.8, 1, 1.25]. To make the scale more compact, each aspect ratio has 5 different scales as [20, 21/5, 22/5, 23/5, 24/5], with a higher scale density, as much as possible to cover all lung nodules.

The evaluation index used in training is mAP (mean average precision), which is also the most commonly used model evaluation index for target detection. Since only one type of target object is lung nodules in this paper, it is only necessary to calculate the average accuracy of lung nodules, where AP is the area under the accuracy and recall curve (PR curve). The initial learning rate used for training is 1*e* − 4. Since each Layer will have more inputs, the number of channels in each layer can be reduced, the feature utilization rate is higher, and the overall calculation will be less than ResNet's feature for the same number of connections. When the model no longer improved for two consecutive training cycles, the learning rate is attenuated, and the attenuation factor is 0.1. After 100 training cycles, the model with the best result is selected. Two data sets were used to train the same detection network, and the data were the data after the rib suppression treatment and the original image of the chest radiograph.

## 3. Result Analysis

### 3.1. Performance Analysis

The self-attention model highlights the semantic difference of the intermediate feature map at each image scale, and then the attention units at different scales can respond to the foreground content of the image. Therefore, this paper integrates the self-attention model into the previous in the 2D V-Net network, and the schematic diagram is shown in Figure 5. In the jump connection, the feature map of the encoder first taken as XL of the self-attention mode. After using the self-attention model to improve 2D V-Net, this paper trains it on the data set, based on the same hardware configuration and software environment, and the segmentation results are shown in Figure 5, which can be seen in the improvement of 2D U-Net. Afterwards, the edge segmentation of CT image segmentation of the new coronary pneumonia is more refined than before, with loss values of 0.0021 and 0.0025 on the training and validation sets, and 0.9834 and 0.9935 of IOU, respectively. And the training time has also been reduced. The original 2D V-Net training time was 46640 seconds, and the training time after adding the self-attention model was 41744 seconds, a reduction of 5.76%.

The article "CT Image Analysis and Clinical Diagnosis of New Coronary Pneumonia Based on Improved Convolutional Neural Network" was published in 2021. Journal: Comput Math Methods Med.

By using the traditional segmentation method and deep learning-based segmentation method, the new-type coronary pneumonia CT image is subjected to binary segmentation of the new coronary pneumonia region, and the results of the level set segmentation are used as the labels for the neural network U-Net and V-Net training, and the original image is simultaneously enhanced with data to expand the data volume. From the segmentation results shown in Figure 6, V-Net performs better and more efficiently than U-Net. Also, this chapter improves 2D V-Net based on the self-attention model. The improved model can more finely segment the target edge, effectively improving the performance of the model. The segmentation results in this chapter will be used for subsequent image diagnosis and three-dimensional reconstruction. Therefore, accurate segmentation results lay the foundation for subsequent work.

In this study, multiple semantic attributes are used as the source task, and multilevel correlation transfer learning is used to assist in the diagnosis of the pathological benign and malignant of pulmonary nodules. First, we use first-order association transfer learning to see which source tasks can better support the pathological diagnosis, then through all the tenth-order transfer learning to find the source task that makes the diagnosis of benign and malignant lung nodules the best. Finally, we compared the multilevel correlation migration method with existing methods and the subjective classification performance of radiologists. We use accuracy, area-under-curve (AUC) score, and Macro-F1 score as evaluation indicators, as shown in Figure 7.

The article "CT Image Analysis and Clinical Diagnosis of New Coronary Pneumonia Based on Improved Convolutional Neural Network" was published in 2021. Journal: Comput Math Methods Med.

Figure 7 shows the performance of first-order transfer learning-assisted diagnosis of pathological benign and malignant pulmonary nodules on accuracy and Macro-F1 indicators. We sorted the contents in Figure 7 by Macro-F1 from small to large for easy comparison. From Figure 7, in the ten semantic source tasks, “text” is used in accuracy, AUC, and Macro-F1 in the first-order transfer learning to assist in the diagnosis of pathological benign and malignant lung nodules. The above performances are the best, indicating that the “text” feature has very important and valuable feature information for the diagnosis of pathological benign and malignant lung nodules. In the first-order migration experiment, the semantic degree (mal) as the source task feature migrated to “pathological benign and malignant (ppm).” Since the semantic malignancy attribute is a doctor's subjective judgment on the malignancy of lung nodules, especially when making a malignant judgment on lung nodules, general doctors tend to conservatively estimate, which may lead to a high misjudgement rate; in the LIDC-IDRI data set, the doctor's misjudgement rate of benign and malignant lung nodules is as high as 28.56%. In our experiments, it was confirmed that using semantic benign and malignant attributes as the source task of transfer learning is not the best choice.

### 3.2. Forecast Results Analysis

We initialize the model with the optimal RetinaNet model trained as a parameter, and then when the data is enhanced, no other expansion methods that may change the location information are used except horizontal symmetry, because in this network, we use the location and scale information. It is not suitable for data expansion through operations such as rotation, translation, and scaling. At the same time, during training, we fixed the network parameters of ResNet in front of the network and only trained the feature pyramid and the parameter weights of the classification and regression subnetwork parts. The selection of hyperparameters for training is the same as when training RetinaNet, and the network with the highest mAP was also selected for comparison. To generate the FROC curve, we selected different score thresholds to output the test results, and then based on the test results, respectively, we calculated the sensitivity under different thresholds; the average false-positive rate and the specific statistical data are shown in Figure 8 This generates the FROC curve.

Finally, the FROC curves of the two models are shown in Figure 8. We can see from the results that the overall FROC curve of LSFNet is above the original RetinaNet model. This shows that the improvement made in this paper for the detection of lung nodules is effective. This is because the points 0.9 and 0.95 are special in nature. Then, to show the difference in effect more intuitively, we select two points with a sensitivity of 0.85 and 0.97 from the curve for specific comparison, as shown in Figure 9.

The article "CT Image Analysis and Clinical Diagnosis of New Coronary Pneumonia Based on Improved Convolutional Neural Network" was published in 2021. Journal: Comput Math Methods Med.

As can be seen from Figure 9, when the sensitivity is the same, the method in this paper can bring a lower false-positive rate. Next, we select one of the cases from dataset A and show the detection results of the two models separately. The sample original image and the labeling situation are shown in Figure 9. This chest radiograph has only one lung nodule, but there are many highlighted areas in the picture, which are easily mistaken as lung nodules. To ensure that the lung nodules are correctly found, it is also to more easily verify that the method proposed in this article can effectively reduce false positives. For the number of samples, we set the threshold to 0.01, so that there will be some false-positive samples in the test results.

### 3.3. Model Diagnosis and Result Analysis

The input of the generator is a set of random noise. The generated result is judged by the discriminator, and the discriminated result is returned to the generator. Because the new coronary artery pneumonia area is smaller than the background area, to reduce the influence of the background area, the image with the initial size of 512 × 512 is cropped and scaled, and the size becomes 128 × 128. Using the same data, DCGAN, WGAN-GP, and PGGAN were trained separately. The implementation details are shown in Figure 10. The generated new coronary pneumonia images are shown in Figure 10. It can be seen that the results generated by WGAN-GP and PGGAN are better than those of DCGAN. Better yet, although DCGAN has a good network framework, the gradient disappears easily during the training process, which is not easy to train. For WGAN-GP and PGGAN, the former is a lightweight network structure, the training process is stable, and there is no need to balance the training times of the generator and the discriminator. The latter is due to the progressive training method, in the same hardware and software environment. Next, the training time is about five times that of the former.

Based on the above image diagnosis process, we first add a mask to the new coronary artery pneumonia area, as shown in Figure 11, and then use it as the input of the generation network, because the model has been trained at this time, that is, the model has saved the information of the generated image; for the image model with a mask added, the mask area will be filled with appropriate and contextual information to make it more consistent with the content of other areas, which is achieved by the loss function. Finally, when the loss function converges, the mask area is filled, that is, the final diagnosis image is obtained, as shown in Figure 11.

The article "CT Image Analysis and Clinical Diagnosis of New Coronary Pneumonia Based on Improved Convolutional Neural Network" was published in 2021. Journal: Comput Math Methods Med.

For the evaluation of the image quality after diagnosis, the paper chooses the largest mean difference, which was first proposed for the two-sample detection problem to determine whether the two distributions are the same. If the value is small enough, the two distributions are considered the same; otherwise, they are considered different. At the same time, this value is also used to determine the similarity between the two distributions. This article uses it to measure the similarity between the original image and the image after diagnosis. KMMD was used for image diagnosis based on WGAN-GP. It is 0.001084, which indicates that the model is effective in diagnosing the missing image area. Volume rendering and surface rendering are two methods of three-dimensional reconstruction. Volume rendering is the direct projection of voxels onto the monitor screen, so it is also called direct rendering; surface rendering is the use of geometric figures to usually fit the target surface for triangular patches. It can also be called indirect drawing. Among them, the better algorithms are the ray casting algorithm and the moving cube algorithm. The accuracy of our model has improved by about 5% compared to the comparative model.

The basic principle of the ray casting algorithm is to emit a ray from each pixel on the screen along the line of sight. If the ray passes through the volume data, it is sampled at equal intervals along the ray direction, and the color of each sampling point is cumulatively calculated by interpolation value and opacity, when the light has passed through the voxel space or reached the set opacity, the projection ends; then, the color values and opacity of the sampling points on each ray are synthesized in order, to obtain the pixels of the projection plane. In the attribute value, this method belongs to volume rendering, which is easy to achieve a good rendering effect and is widely used. First input the original data, read a series of two-dimensional images into memory, construct volume data, and perform preprocessing operations on it. Then, select the appropriate conversion function to convert the scalar values of the volume data to color and opacity from the screen. During the process of the light passing through the entire image sequence, the image sequence is sampled to obtain color information and opacity. Finally, the image plane is rendered according to color accumulation.

The article "CT Image Analysis and Clinical Diagnosis of New Coronary Pneumonia Based on Improved Convolutional Neural Network" was published in 2021. Journal: Comput Math Methods Med.

The moving cube is a classic algorithm for surface rendering and the basis of all voxel-based surface rendering algorithms. The algorithm treats the surface of an object as a closed gray-scale isosurface. If the gray-scale value of the voxel is less than the gray-scale value, then the voxel is located outside the isosurface, and accordingly, if the gray value of the voxel is greater than the gray value, then the voxel is located inside the isosurface. According to the relationship between the data values of the eight vertices of each cube unit and the given data value of the volume data, the algorithm finds the equivalent points on the twelve sides of the cube unit and then connects the equivalent points with triangles to form the isosurface. The specific approach is as follows: First, for volume data, place it in a cube that can be surrounded, then each cross-section parallel to the horizontal plane is a CT image, and then, divide the cube into small cubes, that is, voxel, used for resampling in three-dimensional space, that is, to determine whether the eight vertices of the small cube are inside the target. If a vertex is inside the target object, then the vertex is marked as 0; otherwise, it is marked as 1. The judgment method is to set a threshold, compare the pixel value of the image with it, and determine the state of the vertex. Next, determine the state of the eight vertices according to the picture. There are a total of 256 cases in the arrangement and combination. For each case, some isosurfaces can be generated in the small cube. After obtaining the isosurfaces, calculate the corresponding method.

## 4. Conclusion

In this paper, the U-Net series neural network and the improved 2D V-Net are used to segment the new coronary pneumonia CT images to separate the vertebral body region from other regions. It has good robustness and solves the image noise and tissue incompatibility. Evenness and other issues avoid the defects of traditional image segmentation method of poor edge segmentation. The model used for lesion detection is a network model based on the target-detection task. However, the accuracy requirements of medical images are higher, and a better model is needed; for the diagnosis of the new coronary pneumonia model, consider the spatial information of the new coronary pneumonia and the new coronary pneumonia; the diagnosis of the image can increase the feature information of the upper and lower CT slices; in this paper, based on the target-detection framework Faster RCNN, the feature extraction of the new coronary pneumonia tumor image is performed to obtain a higher-level expression of the image, predict the tumor lesion location, and determine the location of the tumor. Detection and positioning can provide support for doctors' further diagnosis.

The article "CT Image Analysis and Clinical Diagnosis of New Coronary Pneumonia Based on Improved Convolutional Neural Network" was published in 2021. Journal: Comput Math Methods Med.

## Figures and Tables

**Figure 1:** Improved convolutional neural network.

**Figure 2:** Data enhancement process.

**Figure 3:** U-Net framework and specific parameter settings in this article.

**Figure 4:** Performance comparison of lung suppression model.

**Figure 5:** CT images of original new coronary pneumonia and 2D V-Net and improved segmentation results.

**Figure 6:** Loss and IOU curves of the training set and validation set.

**Figure 7:** The performance of first-order transfer learning-assisted diagnosis of pathological benign and malignant pulmonary nodules on accuracy, AUC, and Macro-F1 indicators.

**Figure 8:** Comparison of FROC curve of data set A.

**Figure 9:** Comparison of experimental results of data set A.

**Figure 10:** WGAN-GP model training results.

**Figure 11:** Image diagnosis results.

**Table 1:** Distribution of samples of subordinate subclasses of the nine semantic attributes of novel coronary pneumonia.

Semantic attributes	Number of subclasses	Sample distribution of each subclass
Leaf	8	5
Roundness	7	4
Glitch	10	3
Detail	10	6
Texture	1	4
Edge	9	10
Malignancy	10	1
Internal structure	2	3
Calcification	7	5

## Data Availability

Data sharing not applicable to this article as no datasets were generated or analyzed during the current study.
